# Change of Levels of NGF, ACTH, and AVP in the Cerebrospinal Fluid after Decompressive Craniectomy of Craniocerebral Injury and Their Relationship with Communicating Hydrocephalus

This article has been retracted.

**DOI:** 10.1155/2021/1519904

**Published:** 2021-10-27

**Authors:** Liang Wang, Shuangbo Fan, Zhenping Zhao, Qian Xu

**Affiliations:** Department of Neurosurgery, Ningbo City Zhenhai District People's Hospital, Ningbo, Zhejiang 315200, China

## Abstract

In recent years, the incidence of craniocerebral trauma has increased, making it one of the important causes of death and disability in neurosurgery patients. The decompressive craniectomy (DC) after severe craniocerebral injury has become the preferred treatment for patients with severe craniocerebral injury, but the incidence of postoperative hydrocephalus has become a difficult problem in clinical treatment. This study observed the changes of nerve growth factor (NGF), adrenocorticotropic hormone (ACTH), and arginine vasopressin (AVP) levels in the CSF after DC in patients with craniocerebral injury and analyzed the relationship between the three indicators and communicating hydrocephalus. The results showed that the levels of NGF, ACTH, and AVP in patients with cranial injury after DC were significantly higher than those in healthy subjects, and subdural effusion, traumatic subarachnoid hemorrhage (tSAH), and the levels of NGF, ACTH, and AVP in the CSF were independent risk factors for communicating hydrocephalus. Monitoring the levels of NGF, ACTH, and AVP is of great significance for clinicians to judge the occurrence of traffic hydrocephalus, evaluate the prognosis of patients with craniocerebral injury after DC, and guide clinical treatment.

## 1. Introduction

Craniocerebral injury is the most common cause of death and disability in surgical patients [1]. In recent years, with the development of China's economy and urbanization, the traffic accidents have grown immensely, and the incidence of craniocerebral injury has also increased. DC is an effective surgical procedure for reducing intracranial pressure [2]. With the promotion of this surgical procedure, the mortality of patients with severe craniocerebral injury has decreased [3]. However, postoperative complications tend to occur, affecting the prognosis of patients. Communicating hydrocephalus is one of the postoperative complications of DC induced by CSF malabsorption caused by the increase of CSF protein and the inflammatory viscosity of arachnoid particles [4]. Some studies have confirmed that DC is one of the risk factors for communicating hydrocephalus, but the mechanism is still unclear [5]. It is important to clarify the potential molecular mechanism and risk factors for communicating hydrocephalus after DC for head injury and to improve patient outcomes.

Nerve growth factor (NGF) belongs to the neurotrophic family and plays an important role in maintaining the survival, repair, and regeneration of neurons. Its abnormal expression is considered as an important marker of brain tissue injury [6]. Craniocerebral injury can affect the function of the hypothalamic-pituitary axis indirectly or directly. Therefore, there are some studies suggesting that the measurement of adrenocorticotropic hormone (ACTH) in patients can determine the degree of injury and treatment effect. Arginine vasopressin (AVP) is one of the neuroendocrine hormones secreted by the hypothalamus [7]. It can be involved in the development of secondary injury such as brain edema and has certain correlation with the prognosis of acute craniocerebral injury [8]. This study examined the changes of NGF, ACTH, and AVP levels in patients with BRAIN injury AFTER DC and analyzed the relationship between NGF, ACTH, and AVP levels and traffic-induced hydrocephalus, so as to explore the value of these three indicators in evaluating the prognosis of patients with craniocerebral injury.

## 2. Materials and Methods

### 2.1. General Data

A total of 102 patients with craniocerebral injury who underwent decompression of a large bone flap in our hospital from August 2018 to August 2020 were selected as the study group, including 56 males and 46 females, with an average age of (46.32 ± 9.84) years.

In addition, 90 healthy patients without disease who were admitted to our hospital for lumbar puncture at the same period were selected as the control group, including 49 males and 41 females, with an average age of (47.36 ± 9.25) years. There was no difference in gender and age between the study group and the control group, with comparability (*P* < 0.05).

### 2.2. Inclusion Criteria

All patients with craniocerebral injury were diagnosed as craniocerebral trauma by head CT, CSF routine biochemistry, and clinical manifestations and admitted to hospital within 24 hours after injury.

### 2.3. Exclusion Criteria

Patients with severe systemic infection, patients with a history of thalamic, vertical body, and other neurological disorders, patients with serious injury of other organs or parts, patients with a history of severe acute or chronic illness, patients older than 60 years of age, pregnant or lactating women, and patients who failed to be followed up.

### 2.4. Detection Methods NGF, ACTH, and AVP Level

CSF samples of the study group were collected by lateral ventricular CSF drainage. The CSF samples of the control group were obtained by lumbar puncture. After obtaining the samples, the cell tissues and blood cells were removed by high-speed centrifugation at low temperature after 500 kU/mL aprotinin treatment and stored in a refrigerator at −80°C for further examination.

NGF was determined by Enzyme-Linked ImmunoSorbent Assay (ELISA), and the kit was purchased from Shanghai Waran Biotechnology Co., LTD. According to the instructions of the kit, the optical density at 450 nm was read by using the microplate reader.

The ACTH and AVP levels of CSF were detected by radioimmunoassay. The kit was purchased from DSL, the US, and the instrument was a *γ* counter from DPC, the US. All operations were carried out according to the kit instructions, and all samples were set up double holes and detected in the same batch. At the same time, all samples were tested with serial double-blind.

### 2.5. Assessment Criteria and Data Collection of Communicating Hydrocephalus

Assessment criteria of communicating hydrocephalus [9]: (i) Headache, gait instability, urinary incontinence, mental retardation, and other symptoms that appeared within 3 months after operation. (ii) The head CT and MRI showed that the ventricle system was enlarged to varying degrees, including the following: the lateral ventricle and the third ventricle were round and blunt, and Evan's index >0.3; the periventricular areas such as the frontal and occipital angles of the lateral ventricle showed low-density edema on CT or high-signal edema on T2WI MRI; and the temporal horn of the lateral ventricle was enlarged to varying degrees. According to the occurrence of traffic hydrocephalus, all patients were divided into a communicating hydrocephalus group and noncommunicating hydrocephalus group.

We checked the hospital's medical records system and collected the patient's age, gender, type of craniocerebral injury (closed or open), CSF leak, epidural hematoma, and ventricular hemorrhage, subdural fluid accumulation, traumatic subarachnoid hemorrhage (tSAH), cerebrospinal fluid protein levels, and the Glasgow Coma Scale (GCS), Galveston Orientation and Amnesia Test (GOTA), and functional independent measure (FIM).

### 2.6. Statistical Methods

All data were processed with SPSS 22.0 statistical software, and GraghPad prism 8 was used to make statistical graphs. Measurement data are expressed as mean ± standard deviation ($\bar{x}$ ± *s*), an independent-sample *t*-test is used for comparison between groups, count data are expressed as [*n* (%)], and the chi-square (*χ*^2^) test is performed. Multiple logistic regression analysis was used to analyze the independent risk factors of communicating hydrocephalus after DC. The difference is statistically significant when *P* < 0.05.

## 3. Results

### 3.1. Comparison of NGF, ACTH, and AVP Levels between the Study Group and the Control Group

The levels of NGF, ACTH, and AVP in the study group were higher than those in the control group, with statistical significance (*P* < 0.05, Table 1).

### 3.2. Communicating Hydrocephalus after DC in 102 Patients with Craniocerebral Injury

By the end of follow-up, 31 of the 102 patients had communicating hydrocephalus, and the incidence of communicating hydrocephalus was 30.39%.

### 3.3. Single-Factor Analysis of Influencing Communicating Hydrocephalus after DC of Craniocerebral Injury

There were no significant differences in age, gender, type of craniocerebral injury, GCS, and GOTA score between patients with and without communicating hydrocephalus (*P* > 0.05). There were statistically significant differences in CSF leak, epidural hematoma, ventricular hemorrhage, subdural fluid accumulation, tSAH, CSF protein level, FIM score, and the levels of NGF, ACTH, and AVP in the CSF between the communicating hydrocephalus group and the noncommunicating hydrocephalus group (*P* < 0.05, Table 2).

### 3.4. Assignment of Dependent Variables and Independent Variables of Communicating Hydrocephalus after DC in Patients with Craniocerebral Injury

The occurrence of patients with communicating hydrocephalus was taken as the dependent variable, and the factors with significant differences in Table 2 were incorporated into the logistic regression model as independent variables, and the assignment of dependent variables and independent variables is shown in Table 3.

### 3.5. Multivariate Analysis of Communicating Hydrocephalus after DC in Patients with Craniocerebral Injury

Multivariate analysis results showed that subdural fluid accumulation, tSAH, and the levels of NGF, ACTH, and AVP in the CSF were independent risk factors affecting the occurrence of communicating hydrocephalus after DC (*P* < 0.05, Table 4).

## 4. Discussion

Patients with craniocerebral injury have poor overall prognosis, and the study showed that craniocerebral injury can cause irreversible apoptosis of brain neurons by direct external mechanical force [10, 11]. In addition, the stress response caused by injury can also cause neuroendocrine disorders and inflammatory reactions, which seriously harm the physical and mental health of patients [12]. Dc is often used clinically to relieve intracranial hypertension, reduce brain tissue compression, and restore cerebral blood perfusion, which reduces clinical mortality to a certain extent, but it has little effect on the functional outcome and quality of life of survivors, and postoperative hydrocephalus is still a problem that cannot be ignored [13].

Communicating hydrocephalus is a pathological phenomenon of accumulation in the ventricular system and subarachnoid space due to arachnoid absorption disorder or excessive secretion of the CSF [14]. A. R. S. Neto. et al. reported that the incidence of hydrocephalus after decompressive craniectomy was 34% [15]. Also, a retrospective analysis by W. Qiang-ping et al. showed that the incidence of ventricular enlargement and hydrocephalus was 42.2% and 14.8%, respectively [16]. In our study, the incidence of communicating hydrocephalus was 30.39%, which was within the range of the abovementioned incidence of traumatic hydrocephalus. DC was significantly correlated with postoperative hydrocephalus [17, 18]. The reason is that, after decompressive craniectomy, the skull loses its protective effect, the volume in the skull cavity is unstable, and the normal intracranial pressure balance is destroyed, which affects the CSF pressure, deforms the ventricle, affects the hemodynamics, and finally, affects the generation and absorption of hydrocephalus [19].

In this study, subdural fluid accumulation and tSAH were also independent risk factors for traffic hydrocephalus (*P* < 0.05). The reasons are as follows: ①Ventricle enlargement occurred after subdural effusion subsided which can result in hydrocephalus. Also, because the CSF can penetrate into the subdural space from the ventricle, the subdural fluid accumulation and hydrocephalus can exist at the same time, and they can interact with each other [20]. ② Due to the proliferation and accumulation of arachnoid cells resulting in changes in the structure of the arachnoid villi and the thickening, which increases the resistance of the CSF through the arachnoid villi, it cannot smoothly return to the venous sinus, resulting in hydrocephalus [21].

Communicating hydrocephalus can cause mental retardation, urinary incontinence, and difficulty in movement. It is of great significance for clinical treatment to clarify the high-risk factors of the disease and early predict and diagnose the occurrence of communicating hydrocephalus.

Biological studies have shown that the CSF contains cytokines such as interleukin, as well as molecules such as growth transformation factor-*β* (TGF-*β*) and NGF. Among them, NGF is one of the most important bioactive molecules in the nervous system. In the human body, NGF has a nutritional effect on normal nerve cells [22]. It can maintain the survival of sympathetic and sensory nerves, promote the differentiation of nerve cells, determine the extension direction of axons, and play an important role in brain development, nervous system growth, nerve regeneration, and functional recovery [23]. Changes in the levels of NGF in the CSF after craniocerebral injury are considered to be part of the neuronal recovery process. F. Mashayekhi et al. demonstrated by ELISA that the level of NGF in the CSF of hydrocephalus was higher than that of normal CSF, thus suggesting that NGF is not only a major component in human CSF but may also be involved in the pathophysiological process of hydrocephalus [24]. The changes of NGF in the results of this study were basically consistent with those in the previous study. Also, the multivariate analysis results of our study have shown that the levels of NGF in the CSF were independent risk factors affecting the occurrence of communicating hydrocephalus after DC (*P* < 0.05),indicating a close relationship between NGF and the occurrence of traffic hydrocephalus. Monitoring the changes of CSF NGF level after operation may be helpful to determine the occurrence of communicating hydrocephalus.

After craniocerebral injury, the humoral changes mainly include increased release of antidiuretic hormone, activation of the sympathetic adrenal system, and altered secretion of hypothalamic hormone [25]. The destruction of the blood-CSF barrier can increase the secretion of pituitary hormone ACTH and promote the adrenal expression and release of COR through the hypothalamic-pituitary-adrenal regulatory axis, which can improve the body's antistress [26]. In this process, the body can protect itself. However, the occurrence of hydrocephalus will damage the hypothalamus and pituitary and destroy the negative feedback regulation of the hypothalamus pituitary adrenal axis, increase the levels of ACTH and COR, and cause metabolic disorder and immunosuppression. Therefore, the high level of ACTH suggests that the prognosis of patients with craniocerebral injury is poor. The results of this study showed that there was a significant difference in ACTH level between the communicating hydrocephalus group and noncommunicating hydrocephalus group. ACTH was an independent risk factor for communicating hydrocephalus (*P* < 0.05). Therefore, ACTH was a sensitive index to judge communicating hydrocephalus after craniocerebral injury DC.

Neuropeptide AVP is an endogenous active substance. At first, people thought it was only an important factor protecting the nervous system [27]. However, with the development of molecular biology, some scholars found that AVP can regulate the water balance in the body. It is further speculated that AVP can further induce and aggravate hydrocephalus by participating in the water metabolism of brain tissue and increasing the permeability of capillaries in the injured area of the brain [28]. The increase of AVP content in the CSF of patients in this study group may be related to the increase of catecholamine concentration in blood after craniocerebral injury, which promotes the release of AVP. However, because DC cannot effectively correct catecholamine concentration, it causes AVP to continuously act on capillaries in the brain injury area. It may induce the hydrocephalus. In our study, the logistics regression analysis showed that AVP was an independent risk factor for communicating hydrocephalus (*P* < 0.05), which proved that AVP played an important role in communicating hydrocephalus after DC, and detecting its level had certain clinical value.

In a nutshell, the levels of NGF, ACTH, and AVP in patients with cranial injury after DC were significantly higher than those in healthy subjects, and subdural effusion, traumatic subarachnoid hemorrhage (tSAH), and the levels of NGF, ACTH, and AVP in the CSF were independent risk factors for communicating hydrocephalus. Monitoring the levels of NGF, ACTH, and AVP is of great significance for clinicians to judge the occurrence of traffic hydrocephalus, evaluate the prognosis of patients with craniocerebral injury after DC, and guide clinical treatment. [17]

## Figures and Tables

**Table 1:** Comparison of NGF, ACTH, and AVP levels between the study group and the control group.

Group	NGF (pg/mL)	ACTH (ng/L)	AVP (ng/L)
Study group (*n* = 102)	2.35 ± 0.29	124.51 ± 27.09	25.10 ± 9.53
Control group (*n* = 90)	0.52 ± 0.11	56.28 ± 10.36	12.23 ± 3.12
*T*	56.379	22.482	12.243
*P*	≤0.001	≤0.001	≤0.001

**Table 2:** Single-factor analysis of influencing communicating hydrocephalus after DC of craniocerebral injury.

Clinical information	Communicating hydrocephalus group (*n* = 31)	Noncommunicating hydrocephalus group (*n* = 71)	*χ* ^*2*^ */t*	*P*
Age	48.89 ± 4.75	48.13 ± 5.27	0.690	0.492

Gender				
Male	14 (45.16)	42 (59.15)	1.707	0.191
Female	17 (54.84)	29 (40.85)		

Types of craniocerebral injury				
Closed	18 (58.06)	34 (47.89)	0.894	0.344
Open	13 (41.94)	37 (52.11)		

Cerebrospinal fluid leak				
Yes	25 (80.65)	19 (26.76)	25.543	≤0.001
No	6 (19.35)	52 (73.24)		

Epidural hematoma				
Yes	23 (74.19)	20 (28.17)	18.745	≤0.001
No	8 (25.81)	51 (71.83)		

Ventricular hemorrhage				
Yes	28 (90.32)	23 (32.39)	28.964	≤0.001
No	3 (9.68)	48 (67.61)		

Subdural fluid accumulation				
Yes	25 (80.65)	21 (29.58)	22.728	≤0.001
No	6 (19.35)	50 (70.42)		

tSAH				
Yes	22 (70.97)	14 (19.72)	24.817	≤0.001
No	9 (29.03)	57 (80.28)		

Cerebrospinal fluid protein level				
Abnormal	27 (87.10)	28 (39.44)	19.727	≤0.001
Normal	4 (12.90)	43 (60.56)		
GCS (score)	9.94 ± 2.04	10.53 ± 2.01	1.357	0.178
GOTA (score)	71.35 ± 15.36	73.83 ± 14.98	0.763	0.447
FIM (score)	18.13 ± 1.58	19.95 ± 4.37	2.250	0.037
NGF (pg/mL)	2.09 ± 0.31	1.24 ± 0.26	14.309	≤0.001
ACTH (ng/L)	105.38 ± 19.16	84.33 ± 12.69	6.550	≤0.001
AVP (ng/L)	23.17 ± 5.98	15.33 ± 4.32	7.466	≤0.001

**Table 3:** Assignment of dependent variables and independent variables of communicating hydrocephalus after DC in patients with craniocerebral injury.

Variable	The assignment
Dependent variable	
Communicating hydrocephalus	No = 0, yes = 1

Independent variables	
Cerebrospinal fluid leak	No = 0, yes = 1
Ventricular hemorrhage	No = 0, yes = 1
Epidural hematoma	No = 0, yes = 1
Subdural fluid accumulation	No = 0, yes = 1
tSAH	No = 0, yes = 1
Cerebrospinal fluid protein level	Normal = 0, abnormal = 1
FIM	Enter the actual value
NGF	Enter the actual value
ACTH	Enter the actual value
AVP	Enter the actual value

**Table 4:** Multivariate analysis of communicating hydrocephalus after DC in patients with craniocerebral injury.

Factors	*β*	SE	Wald*χ*^*2*^	*P*	OR (95% CI)
Cerebrospinal fluid leak	0.356	0.328	1.595	0.165	9.364 (0.591∼6.456)
Ventricular hemorrhage	0.732	0.325	4.269	0.325	12.569 (0.964∼8.574)
Epidural hematoma	0.895	0.435	2.695	0.123	13.895 (0.685∼7.334)
Subdural fluid accumulation	2.695	0.485	31.521	≤0.01	20.414 (1.595∼3.592)
tSAH	2.636	0.314	30.589	≤0.01	23.848 (1.923∼4.592)
Cerebrospinal fluid protein level	0.359	0.413	0.639	0.522	10.563 (0.495∼2.834)
FIM	1.633	0.352	16.247	≤0.01	15.656 (1.621∼1.953)
NGF	1.848	0.412	18.953	0.024	18.529 (1.952∼2.633)
ACTH	3.153	0.491	39.254	≤0.01	26.591 (1.832∼2.741)
AVP	4.595	0.844	42.592	≤0.01	29.561 (1.262∼2.894)
Constant	−1.566	0.404	14.988	≤0.01	—

## Data Availability

The data used and analyzed during the current study are available from the first author and corresponding author on reasonable request.
